The article "An Optimization Method Based on Be-ACO Algorithm in Service Composition Context" was published in 2022. Journal: Comput Intell Neurosci.

# An Optimization Method Based on Be-ACO Algorithm in Service Composition Context

**DOI:** 10.1155/2022/5231262

**Published:** 2022-11-22

**Authors:** Zhoujie Du, Huaikou Miao

**Affiliations:** ^1^School of Computer Engineering and Science, Shanghai University, Shanghai 200444, China; ^2^Shanghai Key Laboratory of Computer Software Testing and Evaluating, Shanghai 201112, China

## Abstract

With the increasing complexity of users' needs and increasing uncertainty of a single web service in big data environment, service composition becomes more and more difficult. In order to improve the solution accuracy and computing speed of the constrained optimization model, several improvements are raised on ant colony optimization (ACO) and its calculation strategy. We introduce beetle antenna search (BAS) strategy to avoid the danger of falling into local optimization, and a service composition method based on fusing beetle-ant colony optimization algorithm (Be-ACO) is proposed. The model first generates search subspace for ant colony through beetle antenna search strategy and optimization service set by traversing subspace based on ant colony algorithm. Continuously rely on beetle antenna search strategy to generate the next search subspace in global scope for ant colony to traverse and converge to the global optimal solution finally. The experimental results show that compared with the traditional optimization method, the proposed method improves combination optimization convergence performance and solution accuracy greatly.

## 1. Introduction

In order to solve the interoperability between network applications better and improve efficiency of data sharing and storage, web service composition technology came into being. Due to limited functions provided by individual web service, people began to flexibly and quickly combine existing independent web service platforms to achieve data information mutual exchange and integration to meet the needs of different users. With the increasing complexity of users' needs and increasing uncertainty of individual web service in big data environment, service composition becomes more and more difficult. The requirements of web service composition methods and technologies are becoming higher and higher. The existing web services composition optimization methods mainly include traditional optimization methods and intelligent optimization methods, two categories. Traditional optimization methods have disadvantages such as poor scalability and low flexibility, and they have been replaced by intelligent optimization algorithms gradually. The intelligent optimization algorithms have more obvious advantages than traditional optimization algorithms. First, there is no restriction of central control, and individual failure will not affect the solution of whole problem, which ensures that the algorithm has stronger robustness. Second, they are parallel distributed algorithm model and can make full use of multiprocessors. Third, they have no special requirements for continuity of problem definition and have strong expansibility. Fourth, the implementation of algorithm is simple. Intelligent optimization algorithms can make use of task resources to find service combination optimal solution better and improve algorithm overall performance and resource utilization, for example, common intelligent algorithms include genetic algorithm, ant colony algorithm, simulated annealing algorithm, chaos algorithm, fireworks algorithms, and clustering algorithms [1–13]. Wu et al. [1] proposed an improved genetic algorithm variable neighborhood search to solve hybrid flow shop scheduling problem, and enhance local search ability of genetic algorithm. Previous studies [2, 3] combined chaos idea and genetic algorithm to realize population selection and optimization, which improves efficiency of service composition. Lu and Kou [5] proposed a genetic algorithm based on *ε*-dominance multiobjective is used to solve web service composition optimization problem. The calculation result is a set of compromised Pareto optimal solution, providing users with a variety of options. Zhang et al. [6] improved the particle swarm optimization algorithm and its calculation method and introduced a diversification mechanism to avoid the danger of algorithm falling into local optimum. In the study by Zhang et al. [7], a fast and reliable fault-tolerance approach is proposed for service composition in integration networks, that is, an improved particle swarm optimization algorithm is used to implement service compensation when the permanent faults of service arise. Xing et al. [8] proposed a novel mashup service clustering approach integrating K-means and Agnes algorithms (MSCA). Compared with the traditional mashup service clustering approach based on the K-means algorithm, the average precision rate and recall rate of MSCA improved. Huang et al. [9] greatly improved the ability of web service search engines retrieve services by using the K-means algorithm. In the study by Zhang et al. [11], the improved fireworks algorithm was first applied to discrete services combination optimization problem, and Gaussian mutation probability and elite selection strategy were introduced in the modeling process. Zhang and Yang [13] presented Dynamic QoS Data-driven Reliable Web Service Selection (DQoSRSS), which uses mean and standard deviation to portray the benefit and risk of QoS and to improve the accuracy of QoS description. Due to the interference of various uncertain factors such as the complexity, openness, dynamics, and volatility of cloud service loads in Internet environment, a large number of cloud services with the same functionality have appeared on cloud platform. However, most of their quality of service (QoS) is in an uneven state, which cannot meet the needs of users. In order to handle the QoS-aware cloud service composition problem conveniently and efficiently, there are many representative cluster cooperative intelligent algorithms proposed by scholars such as the ant colony optimization (ACO) system of simulate real ant colony collaboration to find optimized path, genetic algorithm (GA) of mimic biological genetic evolution, particle swarm optimization (PSO) algorithm based on the bird cluster foraging activity model, and so on. Liu et al. [14] proposed a double-elite coevolution algorithm based on three different high fitness individuals as the evolutionary core and adopted different evolutionary strategies to improve algorithm search ability. Xia et al. [15] proposed a global optimization algorithm for dynamic updating multiple pheromones. Compared with the original ant colony algorithm and genetic algorithm, it has better performance in solving service composition optimization problems. Liu et al. [16] proposed a multiobjective service dynamic selection optimization algorithm based on global QoS constraints, and the optimal noninferior solution set can be obtained by optimizing multiple objective functions. Wong et al. [17] proposed a bee colony optimization algorithm based on frequency allocation, which has been improved in experiment of solving traveling salesman problem. A hybrid ant colony genetic algorithm is proposed in the study by Ciornei and Kyriakides [18], which proves the feasibility of this algorithm in dealing with global complex optimization problems. Although the above research methods can solve service composition problem to a certain extent, they all have their own shortcomings. For example, the genetic algorithm has poor local search capabilities and unstable solution results; ant colony optimization pheromone accumulation takes a long time at algorithm initial stage and easy to fall into local optimum. Xie et al. [19] proposed a new swarm intelligence algorithm (social cognitive optimization, SCO). Although SCO can be used to deal with the optimization problems of complex continuous functions, it cannot be used to solve discrete service composition problems. In addition to above problem, the optimization accuracy of the ant colony algorithm is higher than that of the BAS algorithm [20]. The BAS algorithm has fewer adjustment parameters and smaller amount of calculation than some traditional heuristic algorithms, and it has strong global optimization ability. We proposed a service composition optimization method that integrates the beetle-ant colony algorithm in this paper. We fuse BAS algorithm idea to reduce the difficulty of parameter selection in the ant colony algorithm, which overcomes ant colony algorithm to fall into local optimum and obtains the optimal service combination. We verify the feasibility and accuracy of the Be-ACO algorithm through experiments finally.

## 2. Related Work

### 2.1. Service Composition

Service composition mainly includes service request, service calculation, service composition, feedback result of request be processed, generating log file and reporting to cloud service platform, and reporting confirmation. The common cloud computing service model is shown in Figure 1.

Generally speaking, cloud service composition divided into following several processes: first, user sends out service request and transmits it to cloud through edge node server; second, cloud control server divides request task into several subtasks and assigns subtasks to different cloud node servers; third, cloud node server returns result to cloud central server after accomplishing assigned subtask; lastly, cloud central server summarizes processing results of all node servers and feeds back it from cloud server to user through edge node server.

In this paper, the nonfunctional Qo S attribute indicators are used to evaluate service composition quality. We evaluate and study Qo S attribute indicators from the aspects of service time *T*, service cost *C*, availability *Av*, reliability Rel, and reputation Rep. The expression is shown in the following formula:

(1) $$\begin{array}{c} QoS=\left\{T\left(S\right),C\left(S\right),Av\left(S\right),Rel\left(S\right),Rep\left(S\right)\right\}\text{.} \end{array}$$

The specific QoS attribute definition, quantization expression, and normalization processing are based on reference [20], and we assuming that *P* is the path of service composition, then

(2) $$\begin{array}{c} QoS\left(P\right)=\left\{T\left(P\right),C\left(P\right),Av\left(P\right),Rel\left(P\right),Rep\left(P\right)\right\}=F_{Seq}\left(T,C,Av,Rel,Rep\right)+F_{Sel}\left(T,C,Av,Rel,Rep\right)+F_{Par}\left(T,C,Av,Rel,Rep\right)+F_{Cyc}\left(T,C,Av,Rel,Rep\right)\text{.} \end{array}$$

The values of *F*_Seq_, *F*_Sel_, *F*_Par_, and *F*_Cyc_ depend on structure of actual execution path of edge service, and *F*_Seq_+*F*_Sel_+*F*_Par_+*F*_Cyc_=1. We use relevant technologies to convert parallel, selection, and circular structures into serial structures to form service composition model expression, as shown in the following formula:

(3) $$\begin{array}{c} \left\{\begin{array}{c} QoS\left(P\right)=\mathrm{Min}\left(\varphi_{1}T\left(P\right)+\varphi_{2}C\left(P\right)+\frac{\varphi_{3}}{Av\left(P\right)}+\frac{\varphi_{4}}{Rel\left(P\right)}+\frac{\varphi_{5}}{Rep\left(P\right)}\right),\\ \varphi_{1}+\varphi_{2}+\varphi_{3}+\varphi_{4}+\varphi_{5}=1, \end{array}\right. \end{array}$$

### 2.2. Ant Colony Optimization Algorithm

Ant colony optimization was proposed in 1991 by Italian scholar Marco Dorigo. It is an intelligent optimization algorithm that imitates ants finding path process. According to scholars' long-term research on ants' living habits, ants can always find a feasible shortest path from the foraging place to ant nest without any external help, and they can search for a new shortest path based on the constantly changing surrounding environment. The ability of ants to search for the best path is achieved by ants emitting volatile secretion pheromone on the path during the foraging process. The pheromone concentration will weaken gradually with the passage of time. The ants will choose a path according to pheromone concentration of each path when they look for path, and the greater the pheromone concentration on path, the more likely the ant will choose the path [21–23].

The ant will select the next hop path according to the size of pheromone concentration on each path. The following formula represents the state transition probability of the *k*-th ant from node *i* to node *j* at time *t*.

(4) $$\begin{array}{c} P_{ij}^{k}\left(t\right)=\left\{\begin{array}{cc} \frac{{\left[\tau_{ij}\left(t\right)\right]}^{\alpha }∙{\left[\eta_{ij}\left(t\right)\right]}^{\beta }}{\underset{s\in {allowed}_{k}}{\sum }{\left[\tau_{is}\left(t\right)\right]}^{\alpha }∙{\left[\eta_{is}\left(t\right)\right]}^{\beta }}\text{,} & j\in {allowed}_{k},\\ 0\text{,} & others. \end{array}\right. \end{array}$$

In formula (4), *τ*_*ij*_(*t*) and *η*_*ij*_(*t*), respectively, represent the residual pheromone and heuristic information, allowed_k_ represent the nodes that are allowed to select by the *k*-th ant at time *t*, *α* represents the information heuristic factor, and *β* represents the expected heuristic factor. The bigger the information heuristic factor is, the faster the algorithm converges, but it is easy to converge prematurely and fall into local optimal solution and the global optimal solution cannot be obtained. However, the bigger the expected heuristic factor is, the more likely the algorithm is to achieve the global optimization, but the convergence speed of algorithm will decrease. Therefore, the convergence speed of the algorithm and global optimization contradict each other.

In order to prevent too much pheromone remaining on the path from making heuristic information ineffective, update remaining pheromones on the path after *M* ants go from starting point to end point. The amount of pheromone at time *t* + *n* can be updated by the following formulas.

(5) $$\begin{array}{c} \tau_{ij}\left(t+n\right)=\left(1-\rho \right)∙\tau_{ij}\left(t\right)+\Delta \tau_{ij}\left(t\right)\text{,} \end{array}$$

(6) $$\begin{array}{c} \Delta \tau_{ij}\left(t\right)=\overset{M}{\underset{k}{\sum }}∆\tau_{ij}^{k}\left(t\right)\text{.} \end{array}$$

In formula (5), *ρ* represents the volatilization coefficient of pheromone on the path; it is to prevent the pheromone from accumulating continuously and make the algorithm fall into local optimization and miss the better solution. The value range of *ρ* is [0, 1), and 1 − *ρ* represents the pheromone residual coefficient on path. Δ*τ*_*ij*_(*t*) represents the increment of pheromone on path (*i*, *j*) after each search is completed, and Δ*τ*_*ij*_(*t*)=0 at the beginning. ∆*τ*_*ij*_^*k*^(*t*) represents the change of pheromone on path (*i*, *j*) after the *k*-th ant search is complete. Marco Dorigo proposed three different pheromone update models based on different pheromone update methods. They are the ant cycle model, ant quantity model, and ant density model.

With research on the ant colony algorithm, scholars found that the ant colony algorithm can also be used in factory scheduling, multitask matching, image recognition, and other issues. The effect of all these applications mainly depends on selection of ant colony algorithm parameters. The parameters of algorithm performance mainly include information heuristic factor, expected heuristic factor, pheromone volatilization coefficient (or pheromone residue coefficient), pheromone strength, and the number of ant, and the setting of these parameters determines algorithm convergence speed, robustness, and effectiveness. Compared with other intelligent optimization algorithms [24–27] such as the wolf colony algorithm, genetic algorithm, and differential evolution algorithm, the ant colony algorithm has advantages as follows: first, the bottom layer of the ant colony algorithm is a parallel search algorithm actually. In search process, each ant is independent of each other, searches forward in parallel, and works together through residual pheromone. Second, the main feature of the ant colony algorithm is positive feedback. The pheromone left by ants on path can guide following ants to choose the path, which can avoid ants selecting the next hop node blindly. Third, the ant colony algorithm has strong universality, will not cause it to fail to converge due to a little error, and can be well combined with other intelligent optimization algorithms to get better performance. The ant colony algorithm has a certain development in different fields based on above advantages, but it also has its own shortcomings. On the one hand, the ant colony algorithm is easy to fall into local optimization and miss the global optimal solution when algorithm converges too fast. On the other hand, if randomness of ant colony algorithm is increased, the global optimal solution can be improved, but this will lead to algorithm convergence speed slowly at same time. Last, the ant colony algorithm does not have a complete mathematical analysis and theoretical foundation, and most of the parameters are derived from a large number of experimental summaries [28].

### 2.3. Beetle Antenna Search Algorithm

As a novel stochastic optimization algorithm similar to PSO, the beetle antenna search (BAS) algorithm is proposed in 2017 by Jiang and Li [29], which has a more concise search strategy based on beetles' foraging behavior. When the beetle is foraging, if the odor received by left antennae is stronger than that on the right, the beetle moves to left; otherwise, it moves to right. Based on this simple principle, beetle can find food easily. We transform beetle antenna search into an optimization problem in n-dimensional space, where *x*_*l*_ is the left antenna coordinate, *x*_*r*_ is the right antenna coordinate, and *d*^*t*^ is the distance from the center of mass to antenna at time *t*. Since the beetle's head orientation is arbitrary, a standardized random vector can be generated from beetle's right antenna pointing to its left antenna. The standardized random vector is shown in the following formula.

(7) $$\begin{array}{c} \overset{⟶}{b}=\frac{rands\left(n,1\right)}{\left\|rands\left(n,1\right)\right\|}\text{.} \end{array}$$

The generated random vector (beetle's right antenna pointing to its left antenna) is shown in the following formula, where *d*_0_ is the constant distance and *η*_*d*_ is the attenuation coefficient of search distance.

(8) $$\begin{array}{c} x_{l}-x_{r}=2\left(\eta_{d}d^{t-1}+d_{0}\right)*\overset{⟶}{b}\text{.} \end{array}$$

At *t* moment, if position of beetle is *x*^*t*^, the coordinates of left and right antenna are shown in the following formula.

(9) $$\begin{array}{c} {x_{l}}^{t}=x^{t}+\left(\eta_{d}d^{t-1}+d_{0}\right)*\overset{⟶}{b,}{x_{r}}^{t}=x^{t}-\left(\eta_{d}d^{t-1}+d_{0}\right)*\overset{⟶}{b}\text{.} \end{array}$$

If odor function is *f* (*x*), the value of left and right antenna are shown in the following formula.

(10) $$\begin{array}{c} \begin{array}{cc} f_{left}=f\left(x_{l}\right)\text{,} & f_{right}=f\left(x_{r}\right) \end{array}\text{.} \end{array}$$

At *t* − 1 moment, if *f*_left_ > *f*_right_, then beetle moving left, and beetle position in next moment is $x^{t}=x^{t-1}+step*\overset{⟶}{b}$; if *f*_left_ < *f*_right_, then beetle moving right, and beetle position in next moment is $x^{t}=x^{t-1}-step*\overset{⟶}{b}$. According to this rule, we use formula (11) to express beetle moving position in next moment.

(11) $$\begin{array}{c} x^{t}=x^{t-1}-step*\overset{⟶}{b}*sign\left(f_{left}-f_{right}\right), \end{array}$$

(12) $$\begin{array}{c} \begin{array}{cc} step=\delta^{t-1}\text{,} & \delta^{t}=\eta_{\delta }\delta^{t-1} \end{array}\text{.} \end{array}$$

So, *δ*^*t*^ represents the *t*-th iteration step size, sign(*x*) represents the symbol function, and *η*_*δ*_ is the attenuation coefficient of update step.

The BAS algorithm has the characteristics of small computation, fast convergence speed, and global optimization high efficiency. However, the local optimal solution cannot be solved effectively, so it is possible to further optimize the global optimal solution. Based on the above research and analysis, we introduce the BAS algorithm on the basis of ACO algorithm and propose a service composition method based on fusing beetle-ant colony optimization algorithm (i.e., Be-ACO) in this paper. The Be-ACO algorithm fully integrates the characteristics of BAS algorithm's global optimization efficiency and ant colony algorithm accurate solution, thereby improving algorithm time efficiency and solution accuracy.

## 3. Service Composition Optimization Method Based on Be-ACO Algorithm

### 3.1. Be-ACO Algorithm Principle

During the search process of the Be-ACO algorithm, the search mechanism of beetle's movement direction and position update is the same as that described in Section 2.3, and ant colony search subspace is determined by direction and position of beetle's next hop. As shown in Figure 2, the beetle current position is *B*, and the positions of previous hop and next hop are *A* and *C,* respectively; then, ant colony next search subspace is the number of nodes covered by circumcircle area of points *A*, *B*, and *C*, which is recorded as *S*_aco_. *S*_aco_ does not include node *C* and nodes have been searched, and *S*_aco_ = 4 can be seen from Figure 2. Then determine the search target of ant colony in search subspace, that is, the node closest to the global target in set of *S*_aco_ is ant colony search target position in subspace and denoted as *P*_best_. By analogy, until the search is completed, an ant colony searched optimal path is the global optimal solution generally.

Assume that the beetle's position coordinates are *A*(*x*_*t*−1_, *y*_*t*−1_), *B*(*x*_*t*_, *y*_*t*_), and *C*(*x*_*t*+1_, *y*_*t*+1_) at moment *t* − 1, *t,* and *t*+1, respectively. At *t*+1 moment, the ant colony search range is a circular area with *O*(*x*_*O*_, *y*_*O*_) as the center and *R* as the radius; there is no need to search the whole space and make the search efficiency improved greatly. According to Cramer's rule, the coordinates of circle center *O* are obtained, as shown in formula (13), and the radius *R* is updated by formula (14).

(13) $$\begin{array}{c} \left\{\begin{array}{c} \begin{array}{c} x_{O}=\frac{\left[\left(C_{1}*B_{2}\right)-\left(C_{2}*B_{1}\right)\right]}{\left[\left(A_{1}*B_{2}\right)-\left(A_{2}*B_{1}\right)\right]},\\ y_{O}=\frac{\left[\left(A_{1}*C_{2}\right)-\left(A_{2}*C_{1}\right)\right]}{\left[\left(A_{1}*B_{2}\right)-\left(A_{2}*B_{1}\right)\right]}, \end{array} \end{array}\right. \end{array}$$

(14) $$\begin{array}{c} R=\left|OA\right|=\left|OB\right|=\left|OC\right|=\sqrt{{\left(x_{t}-x_{O}\right)}^{2}+{\left(y_{t}-y_{O}\right)}^{2}}\text{,} \end{array}$$

*A*_1_, *B*_1_, *C*_1_, *A*_2_, *B*_2_, and*C*_2_ in formula (13) satisfy the following equation.

(15) $$\begin{array}{c} \left\{\begin{array}{c} A_{1}=2*\left(x_{t}-x_{t-1}\right),\\ B_{1}=2*\left(y_{t}-y_{t-1}\right),\\ C_{1}={x_{t}}^{2}+{y_{t}}^{2}-{x_{t-1}}^{2}-{y_{t-1}}^{2},\\ A_{2}=2*\left(x_{t+1}-x_{t}\right),\\ B_{2}=2*\left(y_{t+1}-y_{t}\right),\\ C_{2}={x_{t+1}}^{2}+{y_{t+1}}^{2}-{x_{t}}^{2}-{y_{t}}^{2}. \end{array}\right. \end{array}$$

### 3.2. Be-ACO Algorithm Process

The Be-ACO algorithm flow is shown in Figure 3, and the Be-ACO algorithm main process includes following steps:

① Initialize the algorithm parameters and beetle objective function *f*(*x*), the beetle movement step=*δ*^*t*−1^ (*δ* is constant), and *t* = 0;
② Initialize the starting search position of subspace, set the starting coordinate as (*x*_0_, *y*_0_), and beetle position coordinate is (*x*_*t*_, *y*_*t*_) at *t* moment;
③ Then *t* = *t* + 1, according to the principle of BAS algorithm in Section 2.3, update the position coordinate of beetle, if *t* < 2, return step ③; otherwise, go to step ④;
④ The current position of the beetle is *P*_beetle_ and *f*(*x*_*t*-1_) < *f*(*x*_*t*_), calculate and obtain ant colony search area according to formulas (13) and (14), update the subset size of *S*_aco_ and the target position *P*_best_ that the ant colony will reach in subsearch space; go to next step;
⑤ According to ACO algorithm principle, ant colony completes search and reaches the optimal position *P*_best_ in subspace; if *P*_best_ is consistent with beetle position *P*_beetle_, execute step ⑥; otherwise, return step ③;
⑥ Search is completed, output the global optimal solution.

## 4. Experiment and Analysis

### 4.1. Simulation Experiment Environment and Parameter Setting

The type of experimental computer is HP880G1, ACPI ×64-based PC; processor is Intel(R) Core(TM) i5-4590CPU @ 3.30 GHz 3.30 GHz; random access memory (RAM) is 4.0 GB; system type is win 8 64-bit operation system; simulation software is MATLAB-R2018b.

Target model:

(16) $$\begin{array}{c} F\left(X_{i}\right)=QoS\left(P\right)=\mathrm{Min}\left(\varphi_{1}T\left(P_{i}\right)+\varphi_{2}C\left(P_{i}\right)+\frac{\varphi_{3}}{Av\left(P_{i}\right)}+\frac{\varphi_{4}}{Rel\left(P_{i}\right)}+\frac{\varphi_{5}}{Rep\left(P_{i}\right)}\right)\text{.} \end{array}$$

Parameter setting: *φ*_1_=0.2, *φ*_2_=0.2, *φ*_3_=0.2, *φ*_4_=0.2, and *φ*_5_=0.2.

In our simulation experiment in this paper, ACO algorithm group scale 0–300 and maximum iterations 300, due to 1 < *α* < 5, 1 < *β* < 5, 0.3 < *ρ* < 0.99, 1 < *Q* < 10000 [30], so we set *α* = 2.5, *β* = 2.5, *ρ* = 0.5, *Q* = 5000; PSO algorithm group scale 0–300, maximum iterations 300, inertia weight 0.6, and learning factor 1; BAS algorithm maximum iterations 300, and adjust the initial value of beetle whiskers length, step size, and attenuation coefficient appropriately according to the range of optimization function variables; Be-ACO algorithm group scale 0–300 and maximum iterations 300 and other parameters settings refer to relevant algorithms.

### 4.2. Experiment Results Analysis

In this experiment, in order to prove the performance superiority of the Be-ACO algorithm by our proposal, ACO, PSO, and BAS are selected to compare the convergence, solution accuracy, and time performance of algorithms, respectively, in this paper.

#### 4.2.1. Convergence Performance and Solution Accuracy

Under the same conditions, the convergence comparison between the ACO algorithm and PSO algorithm is shown in Figure 4. It can be seen from figure that the target value tends to be stable with the increase of iteration times, the convergence speed of ACO algorithm is faster than PSO algorithm, and we can also see the target solution accuracy of the ACO algorithm is higher than that of the PSO algorithm from the convergence curve. As we can see from Figure 5 that the convergence speed of the BAS algorithm is much higher than that of the ACO algorithm, but the solution accuracy of the BAS algorithm is much lower than that of the ACO algorithm.

In order to improve the performance of our algorithm, the design of our Be-ACO algorithm draws on advantage of the fast convergence speed of the BAS algorithm. The experimental results in Figure 6 show our Be-ACO algorithm's convergence performance (CP) is higher than that of the ACO algorithm under same iterations, that is, *CP*_*Be*−ACO_ > *CP*_ACO_, Be-ACO algorithm inherits the fast convergence speed of the BAS algorithm, and it uses fewer iterations than that of ACO when they obtain same target value. The experimental results in Figure 7 show BAS algorithm's convergence performance is higher than our Be-ACO algorithm under the number of iterations is small, but as the number of iterations increases, the solved target value of the Be-ACO algorithm is smaller than BAS, and the solving accuracy (SA) is higher than that of the BAS algorithm, that is, *SA*_*Be*−ACO_ > *SA*_BAS_. The Be-ACO algorithm inherits the solving accuracy of the BAS algorithm and it obtains smaller target value than that of BAS.

Through the experimental comparison between Figures 6 and 7, the Be-ACO proposed in this paper inherits the characteristics of BAS fast convergence speed and ACO high solving accuracy, and it overcomes two algorithms' shortcomings, respectively. In order to further verify performance of the algorithm, we also compared it with the PSO algorithm with good convergence and solution accuracy relatively. The results are shown in Figure 8. The experimental results show that when the number of iterations is the same, the target value solved by the Be-ACO algorithm is smaller, that is, the solution accuracy is higher than that of the PSO algorithm. Under the same target value, the Be-ACO algorithm has fewer iteration times, that is, the convergence speed is faster than that of the PSO algorithm.

In order to more intuitively present the performance of the Be-ACO, BAS, ACO, and PSO algorithms in terms of convergence and solution accuracy, the change trends of several algorithms are shown in Figure 9. The results show that the Be-ACO algorithm has obvious advantages over the three algorithms in terms of convergence and solution accuracy.

#### 4.2.2. Time Performance Analysis

The Be-ACO algorithm proposed in this paper, ACO algorithm, and PSO algorithm have a common feature that algorithm convergence speed slows down with the increase of group scale, and the experimental results are shown in Figure 10. The time cost of ACO and PSO algorithm is greatly affected by group scale, and solution rate decreases significantly, while we proposed the Be-ACO algorithm is less affected by group scale relatively, and the solution rate is significantly better than that of ACO and PSO algorithm.

## 5. Conclusion

The existing web services composition optimization methods mainly include traditional optimization methods and intelligent optimization methods. Traditional optimization methods have been replaced by intelligent optimization algorithms gradually because of poor scalability and low flexibility. The intelligent optimization algorithms have more obvious advantages than traditional optimization algorithms, and it can make use of task resources to find service combination optimal solution better and improving algorithm overall performance and resource utilization. Due to the interference of various uncertain factors such as the complexity, openness, dynamics, and volatility of cloud service loads in Internet environment, a large number of cloud services with the same functionality have appeared on cloud platform. However, most of their quality of service is in an uneven state, which cannot meet the needs of users. Based on above problems, this paper proposes a service composition method based on the beetle-ant colony optimization algorithm. The Be-ACO algorithm combines advantages of BAS and ACO optimization algorithm, while it avoids limitations of their own algorithms. BAS does not consider the connection among groups, but ACO focuses on group influence and ignoring individual influence in the search process. The Be-ACO algorithm proposed by us not only has fast global optimization convergence speed but also has good local optimization effect. In solving the optimal solution of service composition, our method has obvious advantages over BAS, ACO, and PSO intelligent optimization algorithms and methods in terms of convergence and solution accuracy. In future research work, we will optimize this method by combining artificial intelligence, study its optimization method for home robots to handle complex tasks in smart homes [31], and improve the computational efficiency of neural networks; we will also combine convolution neural networks (CNNs) that were applied in the field of medical imaging diagnosis [32] and explore the work to improve the training speed and optimization of initialization parameters to ensure the accuracy of medical diagnosis.

## Figures and Tables

**Figure 1:** Cloud computing service model.

**Figure 2:** Schematic diagram of Be-ACO space search.

**Figure 3:** Flowchart of Be-ACO algorithm.

**Figure 4:** Convergence between ACO and PSO.

**Figure 5:** Convergence between ACO and BAS.

**Figure 6:** Convergence between Be-ACO and ACO.

**Figure 7:** Convergence between Be-ACO and BAS.

**Figure 8:** Convergence between Be-ACO and PSO.

**Figure 9:** Convergence trend graph of several algorithms.

**Figure 10:** Comparison of algorithm efficiency with different group scale sizes under same conditions.

## Data Availability

The experimental result data used to support the findings of this study are included within the article.
